The article "Mesenchymal Stem Cell Therapy for Alzheimer's Disease" was published in 2021. Journal: Stem Cells Int.

# Mesenchymal Stem Cell Therapy for Alzheimer's Disease

**DOI:** 10.1155/2021/7834421

**Published:** 2021-09-01

**Authors:** A. E. Hernández, E. García

**Affiliations:** Facultad de Ciencias de la Salud, Universidad Anáhuac México, Mexico

## Abstract

Alzheimer's disease (AD) is a neurodegenerative disease responsible for 60-70% of the 50 million cases of dementia worldwide. It is characterized by neuronal cell death, shrinkage of brain tissue, and progressive cognitive, motor, and behavioral impairment, which often leads to death. Although current treatment has helped improve the patient's quality of life, it has not been able to alter the underlying disease pathology of AD. Studies have shown that mesenchymal stem cells (MSCs)—a group of multipotent stem cells—have the ability to stimulate neuroregeneration and inhibit disease progression. More recently, extracellular vesicles (EVs) from cytokine-preconditioned MSCs have also shown to induce immunomodulatory and neuroprotective effects in AD models. This review will aim to compile pertinent preclinical AD research on transgenic mice as well as clinical trials on MSC-based therapy from diverse sources.

## 1. Introduction

According to the World Health Organization, around 50 million individuals worldwide suffer from dementia [1]. This figure is expected to double every 20 years, until 2050 [2]. The most common form of dementia is Alzheimer's disease (AD) and may be responsible for 60-70% of the cases [1]. AD is a neurodegenerative disease characterized by the accumulation of extracellular amyloid plaques primarily composed of amyloid-beta (A*β*) peptides and intracellular neurofibrillary tangles (NFTs) of hyperphosphorylated tau protein [3]. Alois Alzheimer first described the disease in 1906 when he reported a 51-year-old woman with cognitive disturbances, delusions, disorientation, and other behavioral changes. AD is associated with neuronal cell death, shrinkage of brain tissue, and progressive cognitive, motor, and behavioral impairment, which often leads to death. As of today, disease-modifying treatments capable of altering the underlying disease pathology of AD are not available [4].

Mesenchymal stem cells (MSCs) are a group of multipotent stem cells capable of differentiating into nonmesenchymal lineages [5]. MSCs are considered a very promising approach to stimulate neuroregeneration due to their immunomodulatory properties and high biosafety but also because of their ability to synthetize neurotrophic and proangiogenic factors [6]. In AD, stem cell therapies have attempted to replace neurons that have been impaired or lost. MSC-based therapies have shown potential to restore damaged neural tissue as well as slow disease progression. Although the specific therapeutic mechanism effect of stem cell transplantation is not known, MSC therapy has shown to be an alternative therapeutic approach for neurodegenerative diseases such as AD [5].

## 2. Pathogenesis of AD and Current Treatment

AD is believed to occur when extracellular senile plaques and intracellular NFTs of hyperphosphorylated tau protein accumulate in the brain. These pathological processes cause a series of downstream events that include neurodegeneration with neuronal and synaptic loss leading to macroscopic atrophy [7]. Although the pathophysiology of AD is still subject to debate, the predominant hypothesis known as the amyloid cascade hypothesis predicts that the accumulation and aggregation of A*β* provoke a pathological set of events that ultimately produce what we know as AD [3, 4]. The amyloid precursor protein (APP) is a transmembrane protein that plays an important role in neuronal development, signaling, and intracellular transport [8]. In the central nervous system (CNS), APP can undergo cleavage either by the nonamyloidogenic or amyloidogenic pathway. In the nonamyloidogenic pathway, APP is first cleaved by *α*-secretase secreting the extracellular soluble peptide alpha (sAPP*α*) and an amino acid fragment known C83, which is later cleaved by *γ*-secretase producing a fragment known as p3. On the other hand, in the amyloidogenic pathway, APP is first cleaved by *β*-secretase, secreting the extracellular soluble peptide beta (sAPP*β*) and an amino acid fragment called C99. *γ*-Secretase also participates in this pathway by cleaving C99, producing a 37-49 amino acid residue peptide known as A*β* [4]. The two main isoforms of A*β* are A*β*40 and A*β*42. The only difference between them is that A*β*42 has two extra residues at the C-terminus. Most amyloid plaques in AD consist of predominantly A*β*42 [9]. The accumulation of A*β* monomers, as well as the decreased clearance, causes it to self-assemble and aggregate into oligomers and eventually into highly regular amyloid fibrils, generating plaques that lead to neurotoxicity and dementia [4]. Soluble A*β* and amyloid plaques are thought to induce a series of events like inflammation, oxidative stress, excitotoxicity, and hyperphosphorylation of tau. This is a protein known for stabilizing and assembling neuronal microtubules. In AD, the hyperphosphorylation of tau promotes insoluble filamentous aggregates that are part of the intracellular NFTs characteristic of the disease [10]. Although the amyloid cascade hypothesis establishes that the hyperphosphorylation of tau is a downstream event of A*β* accumulation, it is possible that tau and A*β* act in parallel pathways causing AD and intensifying each other's toxic effects [2]. In addition, neuroinflammation has also demonstrated to play a key role in AD pathological process. Specifically, microglia have shown to be one of the main players orchestrating inflammation. In AD, uncontrolled microglia activity aggravates tau pathology, stimulates the secretion of proinflammatory cytokines, and causes neuronal injury [11]. Lastly, mass neuronal and synaptic loss is also involved in the AD pathological process. Neurodegeneration affects the entorhinal cortex first, and then the subiculum and CA1 hippocampal subregion and basal forebrain networks. In the advanced stages of AD, the temporal lobes are also affected, ultimately spreading through most cortical layers [12].

AD is commonly divided into familial AD (fAD) and sporadic AD (sAD). fAD is associated with early symptoms of onset and affects <5% of all AD patients. This type of AD is caused by mutations in APP, presenilin 1 (PS1), and/or presenilin 2 (PS2) [13]. Presenilin 1 along with presenilin 2 is the catalytic components of the *γ*-secretase enzyme, which as we previously mentioned, cleaves APP into A*β*s of varying lengths [14]. Thus, fAd-related mutations in presenilins alter the *γ*-secretase cleavage site, resulting in the generation of longer and more fibrillogenic A*β* [15]. On the other hand, sAD, which is associated with late onset, represents nearly 95% of patients with AD. sAD is caused by a combination of genetic and environmental risk factors without a documented familial history of AD. The apolipoprotein E4 (APOE4) and the triggering-receptor expressed on myeloid cells 2 (TREM2) have been considered the two major risk factors for sAD [13]. APOE genotypes have a significant impact on the deposition of A*β* to form senile plaques and cerebral amyloid angiopathy (CAA), two main hallmarks of amyloid pathology in AD [16]. Moreover, TREM2 mutations linked to AD generate a loss of TREM2 protein function, which is a receptor primarily expressed by microglia. This mutation affects the behavior of microglial cells, especially their response to A*β* plaques [17].

For both fAD and sAD, the current treatment includes two different types of pharmacological therapy. On one hand, cholinesterase inhibitors (ChEIs) such as donepezil, rivastigmine, and galantamine are prescribed for mild, moderate, or severe AD dementia [18]. ChEIs improve cognitive symptoms by inhibiting the biological activity of acetylcholinesterase and as a result increases acetylcholine levels in the synaptic cleft, a neurotransmitter used by cholinergic neurons which has been shown to improve the function of brain cells [19]. Response rates vary with approximately around one-third of individuals with AD showing no benefit at all and one-fifth having greater benefit. Similarly, about one-third of patients do not tolerate the ChEIs treatment approach because of side effects [20]. Meanwhile, in moderate to severe AD cases, patients are prescribed memantine, which inhibits the N-methyl-D-aspartate (NMDA) receptor and as a consequence may prevent neuron loss, as well as improve symptoms by restoring damaged neurons. In comparison, NMDA receptor antagonists have fewer side effects than ChEIs [18, 20]. Moreover, a nutraceutical, known as Huperzine A, is also used as an alternative treatment; however, it is not regulated by the Food and Drug Administration (FDA). It is important to note that although the current treatment has helped improve the quality of life of patients living with AD when used at the appropriate time, it has not changed the course or rate of decline of the disease [18]. It has a relatively small average overall effect over AD and is not capable of altering the course of the underlying neurodegenerative process [20].

## 3. MSC as an Alternative Treatment

Stem cells are undifferentiated cells that have the ability to self-renew, proliferate from a single cell, and differentiate into different types of cells and tissues. These cells can be grouped into 4 groups according to their origin: embryonic stem cells (ESCs), induced pluripotent stem cells (iPSCs), and fetal and adult stem cells. MSCs are an example of adult stem cells that can be obtained from various tissues including bone marrow, adipose tissue, bone, Wharton's jelly, umbilical cord blood, and peripheral blood [21]. According to the International Society for Cellular Therapy, MSCs are defined by expressing cluster differentiation (CD), CD90, CD73, CD105, and CD44 while not expressing CD45 and CD31 MSCs normal function in the body includes migrating to injury sites and taking part of a reparative process [22]. In comparison to other stem cells, MSCs differentiation potential is superior as they can differentiate into neuronal cells, osteocytes, chondrocytes, or adipocytes when stimulated with certain growth factors. In addition, MSCs also possess a low risk of differentiating into cancer cells and are infrequently immunogenic [23]. The latter is due to not expressing MHC class II and costimulatory molecules [24]. Moreover, MSCs also possess the ability to migrate to injury and hypoxia sites, boosting tissue repair, reducing apoptosis, and promoting angiogenesis [25].

In AD models, the reduction of A*β* plaques, *β*-secretase, and tau hyperphosphorylation as well as the reversal of microglial inflammation, and the stimulation of anti-inflammatory cytokines are among the mechanisms postulated to have a therapeutic effect in MSC therapy. Upregulating neuroprotection and downregulating proinflammatory cytokines have also been shown to have immunomodulatory and anti-inflammatory effects [26]. In addition, MSC excreted neurotrophic factors have been shown to be able to stimulate neurogenesis and synaptogenesis, alter immune cell response through overexpressing neuroprotective cytokines like IL-10, while reducing proinflammatory cytokines such as TNF-*α* and IL-1*β*, increase the phagocytic activity of microglial cells, improve neovascularization, overcome cell death induced by A*β* and tau, reduce oxidative stress and apoptosis, alter autophagy pathways, and decrease plaque size [27]. Secreted MSC neurotrophic growth factors include glial cell-derived neurotrophic factor (GDNF), vascular endothelial growth factor (VEGF), brain-derived neurotrophic factor (BDNF), insulin-like growth factor 1(IGF-1), nerve growth factor (NGF), and fibroblast growth factor 2 (FGF2) [22, 27]. MSCs have also demonstrated to set off immune responses through microglia activation, which as a consequence sets off anti-inflammatory response. They have also revealed to change microglia phenotype from classically activated to alternatively activated, causing a drop in proinflammatory cytokines and a rise of anti-inflammatory cytokines [28]. Moreover, MSCs also enhance nerve regeneration because of their ability to differentiate into Schwann cell-like cells, which are known for promoting regeneration. MSCs have also demonstrated to boost nerve regeneration via secretion of neurotrophic factors that induce axonal growth and stem cell differentiation into myelinating cell lines [25].

However, the specific mechanism effect of stem cell transplantation is still not known. Possible theories include direct cell replacement of injured neural cells, activation of endogenous stem cells, and secretion of neurotrophic and neuroprotective factors to increase cell survival [29]. In this regard, studies have suggested that the paracrine activity could be the key therapeutic mechanism due to research that indicated that secreted substances in MSC-derived conditioned media, rather than cell incorporation, were responsible for the considerable therapeutic effect in both *in vitro* and *in vivo* contexts [24].

## 4. Preclinical Studies

Many animal models of AD have been studied using different species, such as *C. elegans*, *D. melanogaster*, mouse, rat, and nonhuman primates [29]. However, the most used animal models are transgenic mice which overexpress or silence APP, PS1, and PS2 genes associated with fAD. However, these transgenic mice alone have not been able to replicate most of the pathophysiology of AD. With this in mind, a triple transgenic mouse model with modified APP, PS1, and PS2 was generated. However, it is important to highlight that although a triple transgenic mouse is able to produce A*β* plaques and NFTs, the progressive neuronal loss in the hippocampus and other regions of the human AD brain was not found [30, 31]. On the other hand, no animal model is able to nearly resemble the mechanism and progression of the use of sAD, which is a significant restriction given that this type of AD is significantly more frequent than fAD. As a result, many outcomes found in animal models are rarely seen in clinical studies [13]. The latest findings on MSC therapy in transgenic mouse models of AD will be presented in the next section. A summary is provided in Table 1.

The transplantation of Wharton's Jelly mesenchymal stem cells (WJ-MSCs) has been studied in AD mouse models. Lee et al. investigated the stereotactic administration of human WJ-MSCs and their secreted Agouti-related peptide (AgRP) into the hippocampi of 5XFAD mice which improved proteasome activity and reduced the accumulation of ubiquitin-conjugated proteins. The investigators suggest that either WJ-MSCs or AgRP may be used to delay the clinical progression of AD by improving proteasome activity and consequently lowering abnormal protein aggregation [32]. In another study, Xie et al. found that four weeks after transplantation, WJ-MSCs significantly enhanced spatial learning and mitigated memory decline in APP/PS1 mice. In addition, A*β* deposition and soluble A*β* levels were significantly reduced, while anti-inflammatory cytokine IL-10 significantly increased. Proinflammatory microglial activation and proinflammatory cytokines such as IL-1*β* and TNF*α* were also significantly reduced [33]. More recently, a group of researchers evaluated the difference between “prime” and “naïve” human WJ-MSCs. Prime human WJ-MSCs were previously exposed to an AD cell line via a coculture system and “naïve” human WJ-MSCs. Although both showed promising results in reducing cell death, ubiquitin conjugate levels, and A*β* levels, “prime” human WJ-MSCs showed greater results. This suggests that exposure of human WJ-MSCs to an AD environment improves its therapeutic effects [34].

The transplantation of umbilical cord blood-derived mesenchymal stem cells (UCB-MSCs) has also showed promising results in AD mouse models. In a 5xFAD mouse AD model, human UCB-MS mitigated spatial learning and memory deterioration and alleviated the hyperphosphorylation of tau by GAL-3 secretion [35]. In the same regard, Kim et al. demonstrated that recurring intrathecal (I.T.) administration of human UCB-MSCs improves adult hippocampal neurogenesis and synaptic activity through growth differentiation factor-15 (GDF-15) secretion in an AD model [36]. Human UCB-MSCs have also demonstrated potential to attenuate A*β*42-induced synaptic dysfunction by regulating thrombospondin-1 (TSP-1) secretion [37]. In a study using Tg2576 mice, Cui et al. discovered that human UCB-MSC transplantation significantly mitigated cognitive deterioration of AD mice without altering A*β* levels in the hippocampus. They suggest that human UCB-MSCs may enhance cognitive deterioration by reducing oxidative stress and promoting hippocampal neurogenesis [38]. Moreover, Wang et al. demonstrated that resveratrol facilitates UCB-MSC engraftment in the hippocampus and enhances its therapeutic effect [39]. Similarly, Park et al. studied the coculture of UCB-MSCs, WJ-MSCs, and SVZ-derived neural stem cells (NSCs) in an *in vitro* 5XFAD mouse model. Results demonstrated neuronal development and neurite outgrowth and an increased secretion of activin A. This suggests that both MSCs and activin A may be used to improve neurogenesis for cortical regeneration to treat AD [40].

On the other hand, bone marrow-derived mesenchymal stem cells (BM-MSCs) have also been investigated. Intracerebroventricular (I.C.V.) BM-MSCs have shown potential to improve cognitive deterioration in AD model mice by mitigating astrocytic inflammation and synaptogenesis. Exosomal transfer of miR-146a—which accumulates in astrocytes—is suggested by Nakano et al. to be involved in the improvement of cognitive deterioration [41]. In another study, IL-1, IL-2, TNF-*α*, and IFN-*γ* levels were reduced after human BM-MSC treatment [42]. More recently, a group of researchers investigated the effects of BM-MSCs in 3xTg AD mice using serial [18F] florbetaben positron emission tomography to evaluate the changes in A*β* deposits after MSC therapy. Results showed that a reduction of A*β* deposits in AD mice during BMSC treatment could be confirmed by PET. This opens the possibility that noninvasive PET imaging may be used for the evaluation of MSC response in clinical applications [43]. In the same regard, Park et al. demonstrated that a small number of mouse BM-MSCs are able to reach the brain by intravenous (I.V.) infusion, and a greater distribution of BM-MSCs was found in the 3 × Tg-AD mice compared to a control group. In addition, the results showed that brain uptake increased in the AD group, while the control group did not change significantly [44]. BM-MSC systemic administration in APP/PS1 mouse has also shown the potential to reduce pyroglutamate-modified amyloid-beta (pE3-A*β*) plaque size, a potential biomarker for A*β* plaque pathology [45, 46]. The systemic administration of secretomes isolated from mouse BM-MSCs exposed to AD mouse brain homogenates has also been studied. Santamaria et al. demonstrated that the secretome derived from AD-conditioned MSCs can fully replicate the neuroreparative effects previously associated with MSC direct transplantation. Repeated intranasal (I.N.) infusions of the secretome of APP/PS1 fully restored mouse memory and improved the neuropathology in advanced stages of the disease. Preconditioning BM-MSCs to an AD environment showed to be crucial to induce the therapeutic activity of the secretome [47].

The therapeutic effects of adipose tissue, menstrual blood, and amniotic fluid mesenchymal stem cells have also been studied. Zhao et al. studied menstrual blood-derived mesenchymal stem cells (MenSCs) that showed that intracerebral (IC) injection of them improved A*β* plaques, reduced tau hyperphosphorylation, and enhanced the spatial learning and memory of APP/PS1 mice. They also demonstrated that MenSCs were able to increment various A*β* degrading enzymes and decrease several proinflammatory cytokines such as IL-1*β* and TNF-*α*, which as we previously mentioned are associated with an altered microglial phenotype [48]. On the other hand, adipose tissue-derived mesenchymal stem cells (AD-MSCs) showed to improve endogenous neurogenesis in both the subgranular and subventricular zones, reduce oxidative stress, and mitigate cognitive deterioration in APP/PS1 mice [49]. Similarly, human amniotic mesenchymal stem cell (AM-MSC) intrahippocampal transplantation significantly diminished A*β* deposition and improved the spatial learning and memory deficits in APP/PS1 mice. Zheng et al. suggest that improved cognition may be associated with an increment in hippocampal synaptic density and neurogenesis that is regulated by BDNF [50].

Extracellular vesicles (EVs) from cytokine-preconditioned MSCS are also being investigated as a therapeutic approach for AD due to MSCs reporting paracrine activity. EVs such as exosomes and microvesicles are lipid bilayer vesicles secreted by cells into the extracellular space [11, 51]. Lourdo et al. found that mesenchymal stem cell-derived extracellular vesicles (MCS-EVs) regulate the microglia activation and decreases dendritic spine loss in a triple-transgenic 3xTg mouse [11]. Another study showed that I.V. injected exosomes accumulate mainly in the spleen and liver and not in the brain [52]. Therefore, Cui et al. proposed surface-modified MSC-EVs that target the cortex and hippocampus of AD mice by using a specific rabies viral glycoprotein (RVG) peptide to prevent memory deficits in AD. Results showed that RVG-conjugated mesenchymal stem cell-derived exosomes (MSC-RVG-Exo) improved memory deficits, decreased plaque deposition and A*β* levels, and normalized levels of inflammatory cytokines compared to unmodified exosomes [53].

## 5. Clinical Studies

Many clinical trials have been conducted to evaluate the role of MSCS derived from various sources in patients with AD. It is important to note that only a few have been officially completed and have published results. A summary of the clinical trials registered on ClinicalTrials.gov evaluating MSCs for AD treatment can be found in Table 2.

### 5.1. Completed

A phase 1 clinical trial evaluated a single stereotactic brain infusion of human UCB-MSCs in patients with mild-to-moderate AD. 3 subjects received a single low dose infusion (3.0 × 10^6^ cells/60 *μ*L) while 6 subjects received a high dose infusion (6.0 × 10^6^ cells/60 *μ*L). Results showed that a single injection of human UCB-MSCs was safe and well tolerated and did not cause serious adverse effects during the two-year follow-up. However, it failed to produce the same therapeutic effect as seen in animal studies. Kim et al. speculate that the discrepancy between animal and human studies may be related to the Pittsburgh compound B positron emission tomography (PiB-PET), which may not be sensitive enough to detect soluble amyloid or diffuse amyloid plaques in comparison with immunohistochemical staining, enzyme-linked immunosorbent assay, and Western blot used in preclinical studies, which are capable of detecting soluble and insoluble amyloid as well as different types of amyloid plaques. Another reason as to why the human brain did not replicate findings from the animal studies may be due to their AD microenvironment differences. Similarly, preclinical studies rely on xenogeneic transplantation where as human clinical trials rely on allogenic transplantation. Some limitations of this clinical study include the lack of a control group and the small number of participants [54–56].

A phase 1/2a trial evaluated the safety, dose-limiting toxicity, and exploratory efficacy of 3 repeated intraventricular administrations (I.V.T.) of NEUROSTEM® (human UCB-MSCs) versus placebo via an Ommaya reservoir at 4 week intervals in subjects with AD was completed in December 2019. The study was divided into two stages, stage 1 consisted of a dose escalation in which 3 subjects received a low dose (1 × 10^7^ cells/2 mL) and 6 subjects a high dose (3 × 10^7^ cells/2 mL). On the other hand, stage 2, made up by a randomized and multiple-dose cohort parallel design, consisted of 36 individuals, in which 24 subjects received a high dose with the concentration previously mentioned and 12 received placebo. All groups received 3 repeated I.V.T. infusions via an Ommaya Reservoir at 4 week intervals. The study has yet to publish the results [57].

A phase 1/2 randomized, double-blind, placebo-controlled study was completed on 2019. 21 subjects were randomly assigned into the AstroStem (autologous human AD-MSCs) and placebo control groups in a 1 : 1 ratio. Both groups received 9 repeated I.V. infusions at 2 week intervals, however, only 7 subjects completed the AstroStem infusions and 5 the placebo. Results showed 3 serious adverse effects in the AstroStem group including diarrhea, oesophageal, squamous cell carcinoma stage IV, and pulmonary embolism. Other reported adverse effects were open-angle glaucoma, dysphagia, fatigue, infusion site reaction, fall, dehydration, abnormal loss of weight, syncope, and ecchymosis. The changes in ADAS-Cog score from baseline to week 30 in the AstroStem group were 5.9 (6.8) and 3.0 (5.4) in the control group [58].

### 5.2. Ongoing

A phase 1/2a, open-label, which is currently an ongoing schedule to end in February 2022, was designed to evaluate the safety profile of 4 I.V. infusions of autologous adipose-derived mesenchymal stem cells (HB-adMSCs) in 24 subjects as a possible treatment for AD. 4 I.V. infusions were administered on weeks 0, 2, 6, and 8 at a dose of 2 × 10^8^ total HB-adMSC cells. The main purpose was to evaluate the adverse effects of their treatment as well as the ability of HB-adMSCs to alter AD-related inflammation via measuring the levels of tumor necrosis factor-alpha (TNF-a), interleukin-1 (IL-1), interleukin-6 (IL-6), C-Reactive Protein (CRP), and markers associated with amyloid deposition, A*β*40, and A*β*42. Participants will also be evaluated for cognitive deficits determined by changes in standard values of MMSE, ADCS-ADL, Alzheimer's disease Related Quality of Life (ADRQL), Altoida Neuro Motor Index (NMI) for Digital Biomarkers, and Clinical Dementia Rating Questionnaire (CDR) [59].

A phase 1 placebo-controlled clinical trial designed to evaluate the safety and efficacy of Longeveron Mesenchymal Stem Cells (LMSCs) in individuals with AD is currently ongoing.

A single peripheral I.V. infusion was administered in 25 subjects. Group 1 (10 individuals) received 20 million LMSCs (low-dose), group 2 (10 individuals) received 100 million LMSCs (high-dose), and group 3 (5 individuals) received placebo. To evaluate the safety of the infusion, the incidence of any treatment-emergent serious adverse events was assessed within the first 30 days after treatment administration. Preliminary efficacy was determined by changes in standard values for ADAS-Cog, MMSE, NPI, GDS, University of Pennsylvania Smell Identification Test (UPSIT), ADCS-ADL, Quality of Life-Alzheimer's Disease (QOL-AD), blood inflammatory and AD biomarkers, cerebrospinal fluid inflammatory biomarkers, CSF biomarkers of AD, and brain volumetry calculated using MRI at baseline, 2, 4, 13, 26, 39, and 52 weeks' postinfusion [60].

### 5.3. Challenges

Despite all favorable findings found in MSC-AD therapy, this treatment has several limitations. To begin, no animal model is able to fully replicate the entire pathophysiology of the disease. Similarly, most transgenic mice utilized in preclinical studies rely on the expression of fAD mutations, the least frequent type of AD, while most clinical trials consist of patients with sAD. This complicates the translation of fundamental research findings into clinical investigations. The lack of an effective model that can replicate the entire pathophysiology of the disease is one of the biggest setbacks in the search for an effective AD treatment [31].

Human UCB-MSCs are the most often employed MSCs in clinical studies. However, further research is required to determine if this source is truly the most effective. Correspondingly, the number of injections and delivery routes must also be optimized [71]. In this regard, of the only three completed clinical trials, they all used a different delivery route including I.V., I.V.T., and I.C. The most effective and noninvasive route must be used as repeated infusions will be needed considering that NCT01297218 showed that a single infusion of MSCs was not enough to alter the AD pathophysiological process [11, 54]. Furthermore, further research and appropriate assessment techniques are required to prove the absence of adverse effects from MSC treatment on a long-term basis.

In regard to the administration of MSC-EVs, although preclinical studies have shown promising potential therapeutic effects, it has yet to be studied in patients with AD. As of May 31, 2021, only one clinical trial which is currently recruiting participants is set to study the safety and efficacy of exosomes for AD treatment. However, as suggested by Salem et al., some limitations including EVs heterogeneity, isolation, and production techniques need to be assessed first [28].

## 6. Conclusions

Many preclinical trials evaluating MSC treatment in transgenic mouse models of AD have yielded promising therapeutic outcomes. However, this has not been the case with human clinical trials. Although MSC therapy has demonstrated to be safe and tolerable in a single clinical study with published findings, the therapeutic benefit was not replicated. The frequency of unsuccessful clinical trials might be lowered by developing a successful AD model, notably the one for sAD, which accounts for the vast majority of AD patients. This will allow for a more efficient transition from basic research to clinical trials. Nonetheless, we believe that MSC therapy has a promising future and that its paracrine function, in particular, must be harnessed to establish a successful treatment for AD.

## Figures and Tables

**Table 1:** Most recent findings of MSCs in AD transgenic mice.

Cell type	Model	Study design	Findings
Human WJ-MSCs	5XFAD	Injection of WJ-MSCs or AgRP directly into the left hippocampus of 5XFAD mice.	Improves proteasome activity by AgRP. Reduces the accumulation of ubiquitin-conjugated proteins [32].

Human WJ-MSCs	APP/PS1	Injection of WJ-MSCs into the tail vein of APP/PS1 mice.	Improves the spatial learning. Mitigates memory decline. Increases IL-10. Reduces A*β* deposition levels. Reduces soluble A*β* levels. Proinflammatory microglial activation. Reduces IL-1*β* and TNF*α* levels [33].

Human WJ-MSCs	5XFAD	I.V.T. infusion of WJ-MSCs (exposed to an AD cell line) into 5XFAD mice.	Reduces cell death Reduces ubiquitin conjugate levels Reduces A*β* levels [34].

Human UCB-MSCs	5XFAD	Infusion of recombinant human GAL-3 protein and UCB-MSCs into 5XFAD mice.	Improves the spatial learning. Improves memory impairment. UCB-MSCs mitigate hyperphosphorylation of tau through GAL-3 secretion [35].

Human UCB-MSCs	APP/PS1	Coculture of UCB-MSCs with NSCs to identify paracrine factors. Repeated I.T. injections of UCB-MSCs into APP/PS1 mice.	GDF-15 improves endogenous hippocampal neurogenesis and synaptic activity through CSF [36].

Human UCB-MSCs	5XFAD	Coculture of UCB-MSCs with primary hippocampal neurons under A*β*42 peptide treatment to identify paracrine factors. Transplantation of hUCB-MSCs via I.C.V. route.	Mitigates A*β*42-induced synaptic dysfunction by regulating TSP-1 release [37].

Human UCB-MSCs	Tg2576	UCB-MSCs I.V. transplantation into Tg2576 mice.	Improves cognitive function Attenuates oxidative stress Promotes cell proliferation and newborn cell survival Promotes neurons generating Promotes hippocampal neurogenesis Increases expression of Sirt1, BDNF, and SYN [38].

Human UCB-MSCs	Tg2576	UCB-MSCs I.V. transplantation combined with resveratrol into Tg2576 mice.	Better UCB-MSC engraftment in the hippocampus. Improves learning and memory Enhances neurogenesis Alleviates neural apoptosis in the hippocampus [39].

Human WJ-MSCs and UCB-MSCs	5XFAD	Coculture of MSCs with SVZ-derived NSCs from 5XFAD mice.	Induces neuronal development and neurite outgrowth [40].

Rat BM-MSCs	APP/PS1	I.C.V. injection of BM-MSCs into APP/PS1 mice.	Improves cognitive impairment by ameliorating astrocytic inflammation as well as synaptogenesis by increasing the expression of microRNA-146a in hippocampus [41].

Human BM-MSCs	APP/PS1	Tail I.V. injection of BM-MSCs into APP/PS1 mice.	Reduced levels of IL-1, IL-2, TNF-*α*, and IFN-*γ*. Regulates the expression of A*β*-related genes [42].

Mouse BM-MSCs	3xTg-AD	Evaluation of I.V. injected BM-MSCs using serial [18F] florbetaben PET into 3xTg-AD mice.	The reduction of *β*-amyloid deposits during BMSCs treatment could be confirmed by PET [43].

Mouse BM-MSCs	3 × Tg-AD	Infusion of ^111^In-labeled BM-MSCs via I.V. administration into 3 × Tg-AD mice.	The number of BM-MSCs reaching the brain is very small [44].

Murine BM-MSCs	APP/PS1	Injection of BM-MSCs into APP/PS1 mice via the tail vein.	Reduces pE3-A*β* plaque size. Reduces gene expression of TNF-*α*, IL-6, MCP-1, and NGF. Reduces microglial number and microglia size [45].

Murine BM-MSCs	APP/PS1	Single I.V. and repeated I.N. administration of secretome collected from MSCS exposed *in vitro* to AD mouse brain homogenates from APP/PS1 mouse.	A single infusion: Transient memory recovery Improves the inflammatory phenotype of astrocytes. Reduces brain amyloidosis and microglial activation. Repeated infusions: Sustains memory recovery Reduces neuroinflammation Decreases brain amyloidosis Increases neuronal density in both cortex and hippocampus Diminishes hippocampal shrinkage [47].

Human MenSCs	APP/PS1	I.C. transplantation of MenSCs into an APP/PS1 mice.	Improves the spatial learning and memory Mitigates amyloid plaques Reduces tau hyperphosphorylation Increases A*β* degrading enzymes Modulates a panel of proinflammatory cytokines associated with an altered microglial phenotype [48].

Rat AD-MSCs	APP/PS1	Transplantation of AD-MSCs into the hippocampi of APP/PS1 mice with an automated infusion pump.	Reduces oxidative stress Alleviates cognitive impairment Promotes neurogenesis in the SGZ of the hippocampus Increases the number of neuroblasts in the SVZ of the hippocampus [49].

AM-MSCs	APP/PS1	Intrahippocampal transplantation of AM-MSCs into APP/PS1 mice.	Reduced amyloid-*β* peptide (A*β*) deposition and rescued spatial learning and memory Reduced amyloid-*β* peptide (A*β*) deposition and rescued spatial learning and memory Improves the spatial learning and memory. Reduces A*β* deposition Intensifies release of A*β* degrading enzymes Reduces microglia activation. Increases hippocampal synaptic density and neurogenesis mediated by BDNF [50].

MSC-EVs	3xTg	Administration of EVs derived from cytokine-preconditioned MSCs through the I.N. route into 3xTg mice.	Decrease microglia activation. Increases dendritic spine density [11].

MSC-RVG-Exo	APP/PS1 mice	Use of RVG peptide to target I.V. infused MSC-Exo to the brain of transgenic APP/PS1 mice.	Improves cognitive function better than unmodified exosomes. Decrease plaque deposition and A*β* levels. Reduces the activation of astrocytes. Reduces the expression of proinflammatory mediators such as TNF-*α*, IL-*β*, and IL-6. Raises the levels of IL-10, IL-4, and IL-13 [53].

AD-MSCs: adipose tissue-derived mesenchymal stem cells; AgRP: agouti-related peptide; AM-MSCs: amniotic mesenchymal stem cells; A*β*: amyloid-beta; BDNF: brain-derived neurotrophic factor; BM-MSCs: bone marrow-derived mesenchymal stem cells; CSF: cerebrospinal fluid; EVs: extracellular vesicles; GAL-3: galectin-3; I.C.: intracerebral; I.C.V.: intracerebroventricular; I.N.: intranasal; I.T.: intrathecal; I.V.: intravenous; I.V.T.: intraventricular; IFN-*γ*: interferon-gamma; IL: interleukin; MCP-1: monocyte chemoattractant protein-1; MenSCs: menstrual blood-derived mesenchymal stem cells; MSC-EVs: mesenchymal stem cell-derived extracellular vesicles; MSC-RVG-Exo: RVG-conjugated mesenchymal stem cell-derived; NGF: nerve growth factor; NSCs: neural stem cells; pE3-A*β*: pyroglutamate modified form of amyloid-beta; PET: positron emission tomography; RVG: rabies viral glycoprotein; SGZ: subgranular zone; Sirt1: sirtuin 1; SVZ: subventricular zone; SYN: synaptophysin; TNF-*α*: tumor necrosis factor alpha; UCB-MSCs: umbilical cord blood-derived mesenchymal stem cells; WJ-MSCs: Wharton's Jelly mesenchymal stem cells.

**Table 2:** Clinical trials of MSCs in humans with AD.

NCT	Stage	Cell type	Study design	Phase	Participants	Route	Intervention	Findings
NCT01297218	Completed	Human UCB-MSCs	Open-label, single-center study	1	9	1 single I.C. infusion	250,000 UCB-MSCs per 5 *μ*L per 1 entry site, 3 million cells per brain. 500,000 UCB-MSCs per 5 *μ*L per 1 entry site, 6 million cells per brain.	The stereotactic injection of UCB-MSCs into the hippocampus and precuneus is feasible, safe, and well tolerated. However, a single injection of UCB-MSCs was not effective in altering the AD pathophysiological process [54, 55].
NCT01696591	Unknown	Human UCB-MSCs	Long-term follow-up study of NCT01297218	Same as NCT01297218 [56]				
NCT02054208	Completed	Human UCB-MSCs	Double-blind, single-center study	1/2a	45	3 I.V.T. infusions	1 × 10^7^ UCB-MSCs/2 mL 3 × 10^7^ UCB-MSCs/2 mL Placebo	Not yet published results [57].
NCT03172117	Recruiting	Human UCB-MSCs	Long-term follow-up study of NCT02054208	Same as NCT02054208 [61]				
NCT03117738	Completed	Autologous human AD-MSCs	Randomized, double-blind, placebo-controlled, parallel-group comparison study	1/2	21	9 I.V. infusions	2 × 10^8^ AD-MSCs Placebo	Not yet published results [58].
NCT04228666	Withdrawn	Autologous human AD-MSCs	Open-label, nonrandomized study	1/2a	24	4 I.V. infusions	2 × 10^8^ AD-MSCs	N/A [59]
NCT02600130	Active, not recruiting	LMSCs	Randomized, placebo-controlled study	1	33	1 single I.V. infusion	20 million LMSCs 100 million LMSCs Placebo	N/A [60]
NCT04855955	Available	Autologous human AD-MSCs	Single patient emergency expanded access study	N/A	1	N/A	N/A	N/A [62]
NCT02833792	Recruiting	Human MSCs	Multicenter, randomized, single-blind, placebo-controlled, crossover study	2a	40	1 single I.V. infusion	1.5 million MSCs per kilogram body weight Placebo	N/A [63]
NCT04040348	Recruiting	Allogeneic human UCB-MSCs	Prospective open-label study	1	6	4 I.V. infusions	100 million UCB-MSCs	N/A [64]
NCT04388982	Recruiting	Allogenic AD-MSCs-Exos	Single-center, open-label study	1/2	9	24 nasal drip infusions.	5 *μ*g MSCs-Exos/1 mL 10 *μ*g MSCs-Exos/1 mL 20 *μ*g MSCs-Exos/1 mL	N/A [65]
NCT02899091	Recruiting	P-MSCs	Randomized, double-blind, placebo-controlled study	1/2a	24	1 and 2 I.V. infusions.	2.0 × 10^8^ P-MSCs Placebo	N/A [66]
NCT04684602	Recruiting	Human UCB-MSCs	Multicenter, prospective, open-label clinical study	1/2	5,000	1 single infusion via condition-specific route of administration.	N/A	N/A [67]
NCT04482413	Not yet recruiting	Autologous AD-MSCs	Randomized, double-blind, active-controlled study	2b	80	4 I.V. infusions	2.0 × 10^8^ AD-MSCs/20 mL Placebo	N/A [68]
NCT01547689	Unknown	Human UCB-MSCs	Open-label, single-center, self-control study	1/2	30	8 I.V. infusions	20 million UCB-MSCs (0.5 × 10^6^ UCB-MSCs per kg)	N/A [69]
NCT02672306	Unknown	Human UCB-MSCs	Multicenter, randomized, double-blind, placebo-controlled study	1/2	16	8 I.V. infusions	20 million UCB-MSCs per subject (0.5 × 10^6^ UCMSCs per kg) Placebo	N/A [70]

AD-MSCs: adipose tissue-derived mesenchymal stem cells; AD-MSCs-Exos: adipose tissue-derived mesenchymal stem cells exosomes; AM-MSCs: amniotic mesenchymal stem cells; BM-MSCs: bone marrow-derived mesenchymal stem cells; I.C.: intracerebral; I.C.V.: intracerebroventricular; I.N.: intranasal; I.V.: intravenous; I.V.T.: intraventricular; P-MSCs: placenta-derived mesenchymal stem cells; UCB-MSCs: umbilical cord blood-derived mesenchymal stem cells; WJ-MSCs: Wharton's Jelly mesenchymal stem cells.

## Data Availability

No datasets were generated during the current study.
